The article "Utilization of 3D Laser Scanning for Stability Evaluation and Deformation Monitoring of Landslides" was published in 2022. Journal: J Environ Public Health.

# Utilization of 3D Laser Scanning for Stability Evaluation and Deformation Monitoring of Landslides

**DOI:** 10.1155/2022/8225322

**Published:** 2022-07-21

**Authors:** Yanwei Guo, Xiongwei Li, Shangwei Ju, Qifeng Lyu, Tao Liu

**Affiliations:** ^1^Changzhou Vocational Institute of Engineering, Changzhou Jiangsu 213164, China; ^2^School of Environmental and Safety Engineering, Changzhou University, Changzhou Jiangsu 213164, China; ^3^School of Civil Engineering & Architecture, Changzhou Institute of Technology, Changzhou 213032, China; ^4^Jiangsu Urban and Rural Construction College, Changzhou Jiangsu 213147, China

## Abstract

Three-dimensional laser scanning technology can comprehensively and accurately monitor slope deformation. To conduct deformation monitoring and stability evaluation of the Changzhou Shunguoshan landslide, in this paper, the causes of the Changzhou Shunguoshan landslide were analyzed. Consequently, 3D laser scanning technology and the traditional monitoring methods such as data from the total station were compared. The point cloud data provides big data support for landslide deformation monitoring and landslide stability early warning. Meanwhile, the landslide stability was evaluated by analogy with existing studies on slope deformation monitoring data. Results show that the three-dimensional laser scanning monitoring data is similar to the total station monitoring data. The overall deformation of the Shunguoshan landslide is no more than ± 0.0015 m; the deformation of the Liyang slope is less than ±0.09 m, which is far less than the analog slope deformation monitoring data. The slope construction and monitoring process are in a stable state.

## 1. Introduction

In recent years, geological disasters caused by natural or human factors have had significant impacts on the safety of human life and property and the environment [1, 2]. The specific manifestations are collapse, landslide, debris flow, ground subsidence, ground fissure, ground subsidence, etc. As far as China is concerned, from 2018 to 2021, geological disasters occurred frequently, resulting in a large number of casualties and economic losses. How to reduce the damage and safety hazards caused by geological disasters, it is imperative to “improve the comprehensive monitoring, early identification and forecasting and early warning capabilities of multiple disasters and disaster chains” [3]. The geological disasters in recent years are shown in Figure 1.

Due to the diversity of the Earth's topography (large undulating terrain, many mountains, and hills) and the variability of climate and plate movement [4, 5], rainfall or earthquakes reduce the shear strength of soil and rock layers on slopes [6, 7], and landslides have become one of the most frequent disasters in geological disasters. As far as the landslide deformation monitoring technology is concerned, according to the degree of monitoring automation, the current slope deformation monitoring can be roughly divided into two types, namely, conventional engineering deformation monitoring technology and slope informationization/automation monitoring technology (new slope deformation monitoring technology) [8]. Among them, 3D laser scanning technology is one of the most rapidly developing information/automatic displacement monitoring technologies in the past two decades [9]. The current slope information/automatic monitoring technology (new slope deformation monitoring technology) is shown in Table 1.

As a new type of slope deformation monitoring technology, 3D laser scanning technology is superior to the time-consuming and complex traditional conventional engineering monitoring technology. It is featured with fast timeliness, high accuracy, and high spatial resolution [10]. The importance of 3D laser scanning in slope deformation monitoring can not only monitor slope deformation in a timely, effective and comprehensive manner, but also obtain slope deformation data. In addition, it can also play the role of slope disaster prevention and early warning to ensure the safety of people's lives and property. In China, Huang et al. [11] introduced 3D laser scanning technology and applied it to a slope engineering case, which proved its feasibility in slope deformation monitoring and developed rapidly. Subsequently, Chen et al. [12] established a new method for calculating the volume of landslides by using 3D laser scanning technology, which provided a useful tool for subsequent landslide research. Ma et al. [13] introduced it into the landslide physical model test and compared the overall deformation and displacement of landslide monitoring through different methods (e.g., point cloud stacking and comparison, gravity center method, and fitting method).

The introduction of 3D laser scanning technology into engineering cases has gained momentum. The research directions of this field (or landslide) include slope deformation monitoring, landslide volume calculation, refined analysis of landslides, stability evaluation, and disaster prevention and early warning [14–21]. Research on the application of 3D laser scanning technology under different slope types is shown in Table 2.

Through the existing application research and analysis, the research on the principle and point cloud data processing of 3D laser scanning technology tends to be mature, and it can be applied to the actual working conditions of different slope types with certain reliability. And the application in the field of landside has been developed to a certain extent, but there are few researches on landslide deformation monitoring and stability evaluation based on 3D laser scanning.

Therefore, the 3D laser scanning technology is used to monitor the slope deformation of the Shunguoshan landslide in Changzhou, which provides big data support for landslide deformation analysis and hazard assessment. It is compared with the deformation data measured by the total station to achieve complementation with the traditional monitoring method. The point cloud data analysis provides big data support for landslide deformation monitoring and landslide stability early warning, and the landslide stability evaluation is obtained by analogy with existing studies on slope deformation monitoring data.

## 2. Overview of Shunguoshan Landslide

The Shunguoshan landslide is located in Liangzhuangqiao Village, Zhenglu Town, Tianning District, Changzhou City, Jiangsu Province, in the Yangtze River Delta. It is 1.2 km away from Haigang Avenue in the east and 1.3 km away from Shunjiao Road in the west. For the factory building, there is an easy road leading to the factory area. The central coordinates of the landslide area are *X* = 3525946, *Y* = 516114 (Beijing 54 coordinate system), and the central geographic coordinates are 120°10′12.94″ east longitude and 31°51′21.14″ north latitude.

The lithology of the slope is mainly Silurian Maoshan Formation Middle Series quartz sandstone mixed with silty mudstone. The ground angle of the slope is trapezoidal. Landslide 1 (HP1) (see Figures 2 and 3) is located on the southeast side of the survey area. The length along the slope is about 60 m, the elevation of the top of the slope is +47∼+54 m, the elevation of the bottom of the slope is +4 m ∼+6 m, the height difference is 40∼52 m, and the slope is 34°∼42°.

Due to geological structure and engineering activities (mining), the slope on the northeast side of Shunguo Mountain is high and steep. This is coupled with the special structure of the slope (congruent slope) and stratigraphic lithology (quartz sandstone mixed with silty mudstone), local under the action of heavy rainfall (for several consecutive days in March 2018). As a result, the shear strength of the rock mass decreased. The mudstone softened in water, resulting in collapse and landslide geological disasters.

Specifically, the slope aspect is consistent with the stratum dip angle, the slope is a slope-following structure, and the slope surface is high, steep, and empty. The slope body undergoes creep deformation under the action of gravity, and the slope body has horizontal and vertical displacement. The changes of these displacements further stretch and expand the originally developed joints/cracks in the slope, and cracks appear in the slope.

## 3. Principle and Process of 3D Laser Scanning

### 3.1. Principle of 3D Laser Scanning

The 3D laser scanner adopts active laser scanning technology to detect the monitoring target in all directions to obtain precise positioning. The distance *L* is calculated by measuring the phase difference or time difference required for the first laser pulse to travel from the instrument to the monitored landslide surface and return and to measure the horizontal declination angle *α* and elevation angle *β* at the same time. The positioning principle is shown in Figure 4.

### 3.2. 3D Laser Scanning Equipment and Operation Process

In order to carry out 3D laser scanning of the slope, a Leica MS60 scanner is used, and the angle measurement accuracy can reach 0.5”. This measurement adopts 1000 Hz mode for scanning, its ranging accuracy is 300 m/1.0 mm, and the distance is 50 m. The relevant parameters are shown in Table 3. The main process of scanning is shown in Figure 5.

## 4. Data Collection and Analysis

### 4.1. On-Site Data Collection

After the construction of the slope of Shunguo Mountain was completed, two phases of scanning work were completed successively by 3D laser scanning. The status of the slope during the operation period before and after the rainy season was monitored and analyzed, as shown in Figure 6.

The first phase of scanning work was carried out on May 16, 2020. On the afternoon of May 16, the main part of the slope was scanned. The scanning distance was 170 m, and the horizontal and vertical point intervals of the farthest point were 5 mm and 10 mm, respectively. The second scan was carried out on the afternoon of November 28 after the rainy season. The distance, range, and point interval of this scan were basically the same as those on May 16.

### 4.2. Initial Modeling of Slope

The collected original point cloud data of Shunguoshan was filtered and denoised to remove redundant information and noise data. Consequently, the point cloud data was registered, and a solid model was established corresponding to the slope according to the slope shape and point cloud data, namely, the 3D model reconstruction. The detailed process and method are shown in Table 4. The initial modeling of the slope is shown in Figure 7.

### 4.3. Point Cloud Data Analysis

On the afternoon of May 16, 2020, the main part of the slope was scanned, with a scanning distance of 170 m, and the horizontal and vertical point intervals of the farthest point were 5 mm and 10 mm, respectively; the second phase of the scanning operation was carried out on the afternoon of November 28. The scanning distance, range, and point interval are the same as those on May 16. The chromatogram analysis is carried out through the polyworks software superimposed through the two-phase data acquisition. For the specific analysis of the chromatogram, please refer to Figure 8.

A total of 37 displacement monitoring points are arranged in the slope deformation monitoring area, and six monitoring points, J8, J9, J10, J12, J13, and J14, are selected in the scanning area (as shown in Figure 9). The direction and level changes are shown in Figure 10.

Results showed that the three-dimensional laser scanning monitoring data was similar to the total station monitoring data, and the vertical data at points J12, J13, and J14 had an error of 1 mm, which may be related to the actual weather and operation at that time. Among them, the maximum vertical displacement of the laser is 0.0015 m, the maximum horizontal displacement of the laser is 0.0009 m, and the displacement does not exceed ±1.5 mm, indicating that the treated slope is in a stable state. After the rainy season, the slope is still stable, and the slope protection has reached the design target.

We compared the vertical and horizontal monitoring data with the total station as shown in Figure 11.

## 5. Case Analysis of 3D Laser Scanning Monitoring during Slope Construction

The three-dimensional laser scanning monitoring of the Shun Guoshan project was performed during the operation period. In order to examine the applicability of the 3D laser scanning method during the construction period, we carried out the 3D laser scanning construction period monitoring of a slope under construction in Liyang area at the same time, and we carried out a research on the instability risk evaluation of the high slope during the construction period. The Liyang Slope is located in Liyang, Changzhou, on the northwest side of the slope of Shunguo Mountain, about 110 kilometers apart.

### 5.1. Raw Point Cloud Data Acquisition and Initial Modeling

We go to the monitoring site and complete the first on-site application, the collection of raw point cloud data. The collected original point cloud data is filtered and denoised to remove redundant information and noise data. Then the point cloud data is spliced, that is, three-dimensional modeling. The preliminary results are shown in Figure 12.

### 5.2. Analysis of Slope Body Deformation in Area a

Following the second 3D laser scanning, the point cloud data of the first and second scans are superimposed to obtain the analysis effect diagram of the slope deformation point cloud of the second-1st period. The analysis flow chart of area A is shown in Figure 13.

Deformation diagram of slope body in area A (point cloud data chromatogram comparison diagram) is shown in Figure 14. According to the point cloud data, from the analysis of phase 2-1 and phase 3-2 deformation maps, the overall displacement of the slope here is relatively stable, and the deformation is less than ±0.05 m. Although the local fluctuation is large, there is no obvious change. Preliminary finding is that there is no overall slump risk of the slope here. However, the surface layer of the slope, especially the third-level slope, has the risk of local collapse and the fall of weathered rock and soil. Attention should be paid to the follow-up construction process and strengthen construction protection.

According to the observation of phase 4-3, the displacement of the slope surface is relatively stable as a whole. The deformation amount is less than ±3 cm, and there is no obvious local fluctuation and large deformation. Since all the slope excavation has been completed and there is less disturbance, there is no overall risk of collapse of the slope here. However, the subsequent construction process may impact the slope, and it is necessary to pay attention to observation and strengthen protection.

The deformation diagrams of phases 5-4 and 6-5 are analyzed. The displacements of grades 4, 5, and 6 and the slopes of grades 3 and 4 are relatively small, and the overall stability is relatively stable. No obvious construction safety hazards are found. According to different points in the chromatogram, it can be observed that the third-level slope and the first-level slope have an uneven local settlement, and certain support methods should be adopted.

In phase 7-6, the slope displacement is small, the overall is relatively stable, and the difference between the point cloud data and the previous phase is small. There is no obvious construction safety hazard.

To sum up, during the construction process, the maximum deformation of the slope here is not more than ±0.05 m, and there is a certain degree of uneven settlement locally, but the whole is in a stable state. With the progress of construction protection, the state of the slope becomes more and more stable.

### 5.3. Analysis of Slope Body Deformation in Area b

After the third 3D laser scanning of the slope, the schematic diagrams of the point cloud data of the second and third scans were superimposed. The purpose is to obtain the effect diagram of the slope deformation point cloud of the third and second phases. The analysis flow chart of area B is shown in Figure 15.

Deformation diagram of slope body in area B (point cloud data chromatogram comparison diagram) is shown in Figure 16. According to the point cloud data, the deformation maps of phases 2-1 and 3-2 were observed. The displacement of the slope surface was relatively small, the overall stability was relatively stable, and there were no obvious construction safety hazards. However, some points in the chromatogram were selected in phase 3-2, and it can be observed that the slope has uneven settlement and uplift of ±0.1 m, and attention should be paid to later construction and protection.

According to the analysis of the deformation diagrams of phases 4 and 3, the displacement of the fourth, fifth, and sixth slopes is relatively small, the overall stability is relatively stable, and there is no obvious hidden danger of construction safety. However, by clicking on some different points in the chromatogram, it can be observed that the third-level slope has uneven settlement and uplift of ±0.04 m, which is due to the local uneven deformation caused by blasting construction and excavation and unloading of the second-level slope. Certain support methods should be adopted.

In the 5-4th, 6-5th and 7-6th phases, the slope displacement of the slope is relatively stable as a whole, the deformation amount is less than ±0.015 m, and there is no obvious local fluctuation large deformation. Since there is no construction excavation shortly and there is a less artificial disturbance, there is no overall risk of slope collapse here. However, the subsequent construction process may impact the slope, and it is necessary to pay attention to observation and strengthen protection. Phases 7-6 indicate that the excavation below the slope causes less disturbance to the upper part.

In short, during the construction process of this slope, there are local settlements and uplifts with a maximum amount of no more than ±0.1 m and the whole is in a stable state. With the progress of construction protection, there are fewer safety hazards on the slope.

### 5.4. Comparative Analysis of Deformation and Displacement of Each Slope

Three-dimensional laser scanning technology was used to monitor the Shunguoshan slope in Changzhou and the two slopes in Liyang, and the deformation data was obtained through point cloud data processing, which was compared with the data in the previous studies, as shown in Table 5.

It can be observed that the monitoring deformation data of Shunguoshan slope in Changzhou is much smaller than that in the analogy literature [19]. The slope has been designed for slope reduction, load reduction, anchor cable anchoring, stone retaining wall, and greening design and is in a stable state.

Similarly, the monitored deformation data of the two slopes in Liyang are slightly larger than the maximum displacement of Shun over the mountain and far smaller than the monitoring data of the slope deformation in the analogous literature [17, 20]. The slope stability has a certain influence, resulting in deformation, yet it is still in a stable state.

However, the research in this paper has certain limitations. This paper only discusses the application of 3D laser scanning technology in monitoring slope deformation, including horizontal displacement, vertical displacement, and absolute displacement. However, 3D laser scanning can not only monitor slope deformation and displacement, but also perform landslide volume calculation and landslide refinement analysis, which is the focus of future research.

At the same time, 3D laser scanning technology still has certain shortcomings. Its equipment cost is high, and the price of 3D scanning machine is relatively expensive; it is greatly affected by bad weather and cannot operate normally under weather conditions such as heavy fog, heavy rain, and strong wind. Point cloud data also produces a lot of noise, and point cloud data processing is difficult. However, geological disasters such as landslides often occur under the influence of extreme weather. Therefore, how to monitor the slope deformation under extreme weather conditions (three-dimensional laser scanning monitoring) is the focus of future researches.

## 6. Conclusion

Three-dimensional laser scanning was used to obtain the surface displacement of the slope through intermittent monitoring to develop a sloping point cloud data map to examine the stability of the slope. The landslide deformation map was analyzed based on the vertical displacement change and the horizontal displacement change under the splicing of point cloud data. For the slope of Shunguo Mountain that experienced the rainy season, the results showed that the maximum vertical displacement of the landslide was 0.0015 m, and the maximum horizontal displacement was 0.0009 m. The amount of landslides is not more than 0.0015 m, and the landslide is in a stable state. For the same two slopes in Liyang, the maximum displacement of slope A is 0.0323 m, and the maximum displacement of slope B is 0.0889 m, and the slope as a whole is in a stable state.

3D laser scanning can analyze the overall slope and examine it accurately to any point. The data obtained by scanning feature points makes the data of the entire surface have more detailed precision.

Unlike traditional methods, 3D laser scanning monitoring has a certain degree of accuracy, and noncontact measurement points are more digital and information-based. It can complement traditional monitoring methods, improve the efficiency of slope monitoring, and provide data support for slope protection, early warning, and stability assessment.

The slope monitoring method of 3D laser scanning is suitable for slope monitoring during operation as well as slope monitoring during construction. It can be widely used in geological disaster warning and engineering construction projects in the future.

The successful application of 3D laser scanning technology in the deformation monitoring of Shunguoshan slope further demonstrates the feasibility of 3D laser scanning technology, provides a new solution for slope deformation monitoring, and provides future landslide warning and slope stability. The evaluation provides an example and accumulates experience for the popularization and application of advanced slope technology in the future.

## Figures and Tables

**Figure 1:** Geological disasters in recent years.

**Figure 2:** Scene of landslide 1.

**Figure 3:** The trailing edge of the top of the landslide.

**Figure 4:** Principle of 3D laser scanning positioning.

**Figure 5:** Scanning flowchart.

**Figure 6:** Slope data collection site. (a) 2020-5-16. (b) 2020-11-28.

**Figure 7:** The initial modeling of the slope.

**Figure 8:** Point cloud data chromatogram. (a) The first phase. (b) The second term. (c) Point cloud data chromatographic comparison.

**Figure 9:** Layout of displacement monitoring points.

**Figure 10:** Vertical and horizontal displacement variation of 3D laser scanning. (a) Vertical displacement change. (b) Variation of horizontal displacement.

**Figure 11:** Deformation and displacement of the landslide using total station and 3D scanner. (a) Comparisons of vertical displacement. (b) Comparisons of horizontal displacement.

**Figure 12:** Schematic diagram of 3D modeling of slope. (a) Area a. (b) Area b.

**Figure 13:** Process of phase 2-1 deformation diagram.

**Figure 14:** Deformation diagram of slope body in area A (point cloud data chromatogram comparison diagram). (a) Issue 2-1. (b) Issue 3-2. (c) Issue 4-3. (d) Issue 5-4. (e) Issue 6-5. (f) Issue 7-6.

**Figure 15:** Process of phase 3-2 deformation diagram.

**Figure 16:** Deformation diagram of slope body in area B (point cloud data chromatogram comparison diagram). (a) Issue 2-1. (b) Issue 3-2. (c) Issue 4-3. (d) Issue 5-4. (e) Issue 6-5. (f) Issue 7-6.

**Table 1:** Current slope information/automatic monitoring technology (new slope deformation monitoring technology).

Technical method			A brief introduction to the principles of different monitoring methods	Advantage	Disadvantage
“3S” technology	Measuring robot		The measuring robot combines laser technology, communication technology and CCD technology to form a measuring platform integrating target recognition, tracking, automatic sighting, angle measurement, ranging, recording and other technologies, which can accurately obtain unstable targets of slope geology data; the continuous and repeated monitoring of extremely many targets is completed in a short time, and the fully automated geological data measurement is realized	Automation, informatization, strong continuity, and strong data reliability	Higher investment and maintenance costs
	Remote Sensing Technology (RS)		Receive electromagnetic wave information from various geographies on the Earth's surface by satellites, drones, etc. from high altitude or outer space, and scan, photograph, transmit, and process this information, so as to conduct long-distance research on various ground objects and phenomena on the Earth's surface; modern comprehensive technology for control, measurement, and identification	Wide monitoring range, quick access to information, small geomorphological restrictions, strong periodicity, and low investment	Affected by bad weather (heavy rain, strong wind, ice and snow, etc.); the accuracy needs to be improved
	Geographic Information Systems Technology (GIS)		The technology of collecting, storing, managing, processing, analyzing, displaying, and describing the relevant geographical distribution data in the whole or part of the Earth's surface (including the atmosphere) space with computer hardware and software systems	Strong acquisition, analysis, and calculation capabilities	Insufficient models and data structures restrict development
	Satellite Navigation System Technology (GPS)	CORS technology GNSS technology	Use the navigation and positioning signals sent by GPS satellites to carry out spatial resection measurement, determine the three-dimensional coordinates of the ground to be measured, and obtain absolute displacement data and its changes according to the changes of coordinate values in different time periods	Strong continuity, high real-time, three-dimensional, high-precision, automation, informatization	Affected by the environment, which affects the signal strength

3D Laser Scanning Technology			Active laser scanning technology is used to detect the monitoring target in all directions, so as to obtain accurate positioning	Wide range, high precision, and high efficiency	Higher cost, affected by bad weather
Interferometric Radar Technology (InSAR)	DInSAR technology MT InSAR technology		The radar is used to transmit microwaves to the target area and then receive the echoes reflected by the target to obtain the SAR complex image pair imaged in the same target area; if there is a coherence condition between the complex image pairs, the SAR complex image pair can be conjugated to obtain the interferogram by multiplying it; according to the phase value of the interferogram, the path difference of the microwaves in the two imaging is obtained, so as to calculate the topography and small changes of the surface of the target area	Wide range, high continuity, low data volume, low cost	Affected by bad weather, Affected by DEM
Close-up photogrammetry			A measurement technology that uses noncontact data acquisition by processing images such as measurement and interpretation	Low cost, high flexibility, and strong applicability	Photo interpretation accuracy is slightly poor

**Table 2:** Research on the application of 3D laser scanning technology under different slope types.

Slope type	Author (year)	Research content
Open-pit mining slope	Depeng YU et al. (2010) [14]	The three-dimensional laser scanning technology is used to monitor it, and the point cloud data acquisition and processing are used to analyze its deformation characteristics to study the slope's distortion accurately.
	E. Manda Mvula et al. (2019) [15]	The sloping structure is scanned by 3D laser scanning technology, and a comprehensive, reasonable and reliable 3D point cloud structure database is created.
Water conservancy engineering slope	Hu Chao et al. (2015) [16]	Using 3D laser scanning technology to calculate the excavation volume of the slope, a new algorithm for calculating the volume of the excavation body using laser scanning data is proposed.
Mountain slope	Yiheng Pan et al. [17] (2014)	The design, data acquisition, data processing and data analysis of 3D laser scanning monitoring scheme are systematically introduced. From this, the overall deformation characteristics of Ginkgo landslide and the advantages and disadvantages of 3D laser scanning technology in landslide monitoring are obtained.
	Kociuba W et al. [18] (2014)	The application of terrestrial laser scanning (TLS) to accurately model land landforms and quantitatively estimate spatial and temporal transformations can contribute to a better understanding of watershed formation processes.
High road slope	Mengyuan Si, etc. [19] (2020)	Three-dimensional laser scanning technology is used to study its deformation monitoring to evaluate and warn the slope stability
Cliffside	Kuhn, D. et al. [20] (2014)	Using 3D laser scanning technology, high-resolution laser scans of the ground surface (including landslide expansion, spatial and temporal variations) were performed over five years of a cliff, and calculations were performed to quantify the large volumes that lead to erosion processes and slope instability.
High Slope of Domestic Waste Incineration Power Plant	Wenlian Liu et al. [21] (2021)	The spatial distribution and geometric form of argillized interlayers in rock slopes are analyzed and studied by using 3D laser scanning technology.

**Table 3:** Equipment parameters.

Hardware performance indicators	Scan distance	Ranging accuracy	Color image	Control connection	Working environment	Equipment weight (kg)
Parameter value	1.5 m∼1000 m	1 mm + 1.5 ppm	5-megapixel CMOS sensor; onboard 3D point cloud viewing capability, true color point cloud	RS232, USB, Bluetooth®,wlan	IP65	7.7

**Table 4:** Point cloud data slope model reconstruction process and method.

Processing steps	Handling operations	Approach
1	Point cloud data preprocessing	Noise point removal, invalid point cloud data filtering
2	Target localization and registration	It is based on the software's target positioning and converting the station scan data to a unified coordinate system
3	Visual model building	We reconstruct the visualization model of the slope through the point cloud meshing algorithm
4	Point cloud simplification	Simplify the reconstructed model to make the analysis as easy as possible
5	Deformation measurement	The models in different periods are superimposed and analyzed through point cloud superposition to obtain deformation data

**Table 5:** Comparison of the deformation and displacement of each slope.

Monitoring slopes	Maximum vertical displacement (m)	Maximum horizontal displacement (m)	Maximum displacement (m)	Average displacement (m)
Shun crosses the slope of the mountain	0.0015	0.0009		
Si Mengyuan et al. [19] (2020)	0.1027	0.0636		
Liyang Slope A			0.0323	
Liyang Slope B			0.0889	
Yiheng Pan et al. [17] (2014)			1.392	0.0125
Kuhn, D. et al. [20] (2014)			17.32	3.46

## Data Availability

Upon request, the data supporting the conclusion of our study are accessible from the corresponding author.
